RETRACTED

# Pollution halo impact in context of productive capacities, energy poverty, urbanization, and institutional quality

**DOI:** 10.1371/journal.pone.0295447

**Published:** 2023-12-07

**Authors:** Yuqiang Mo, Ghulam Rasool Madni

**Affiliations:** 1 Faculty of Innovation and Design, City University of Macau, Macau, China; 2 Beijing Institute of Technology, Zhuhai, Zhuhai, Guangdong, China; 3 Department of Economics, Division of Management and Administrative Science, University of Education, Lahore, Pakistan; University of Pitesti, Romania; Institute of Doctoral and Post-doctoral Studies, University Lucian Blaga of Sibiu, ROMANIA

## Abstract

The Belt and Road Initiative (BRI) represents a substantial development strategy spearheaded by China. Its central aim is to foster connectivity across a vast geographical area that includes countries spanning Asia, Europe, and Africa. This project played a pivotal role to develop the region on the one side and also raised serious environmental concerns on the other side. There is extensive literature explored the various dimensions affecting the environment in BRI partner countries but there is hardly any study examining the impact of productive capacities, energy poverty, FDI, urbanization, and institutional quality on CO2 emission in the BRI region. Moreover, pollution halo impact is also explored so this study used panel data of 52 nations engaged in the BRI covering time span of 2001–2022 by applying OLS, Difference GMM, System GMM, Cross sectional-ARDL techniques. The results suggest that enhancing productive capacities, FDI and institutional quality significantly reduces carbon emissions in the region, while energy poverty, urbanization and economic growth is linked to higher carbon emissions. Moreover, ‘pollution halo effect’ is proved because of adoption of eco-friendly technologies through foreign corporations lead to reduction in carbon emission. The study advocates for policy measures that emphasize the promotion of productive capacities, the utilization of renewable energy sources, the adoption of practices regarding sustainable urban development, the implementation of efficient institutional structure, and inflow of eco-friendly technology through FDI.

## 1. Introduction

Recently, many problems are rising from global climate change and these problems are threatening both humanity and ecosystems [1]. There are various international frameworks and agreements regarding climate change on a global scale, such as the SDGs, the Paris Agreement, and the 26th Climate Change Conference. In line with the United Nations’ sustainable development goals (SDGs), countries are taking action to achieve their carbon reduction goals [2]. Environmental preservation and climatic changes are closely interconnected with several SDGs outlined by the United Nations. Understanding the links between environmental degradation and SDGs is essential for developing holistic and effective strategies for sustainable development. The SDGs are a set of 17 global goals that aim to address various social, economic, and environmental challenges to achieve sustainable development by 2030 [3, 4]. SDG 7 aims to ensure access to affordable, reliable, sustainable, and modern energy for all. while SDG 13 explicitly focuses on taking urgent action to combat climate change and its impacts. Reducing CO2 emissions is a critical component of SDG 13, and efforts to mitigate climate change contribute to achieving sustainability [5, 6]. In essence, sustainable development aims to harmonize economic progress with habitat preservation, or economic development with the conservation of natural ecosystems [7].

RETRACTED

Environmental degradation is a pressing issue facing humanity presently and primary driver of this degradation is the greenhouse effect, which is attributed to increase in carbon dioxide emissions [8]. These emissions have surged from 280 parts per million (ppm) during the preindustrial period in 18th century to over 400 ppm now [9]. Carbon dioxide emissions are recognized as a significant contributor to environmental pollution [10]. The share of different parts of world in CO2 emissions is shown in Fig 1.

**Fig 1:** Share in global CO2 emissions. Source: Salam and Xu [11].

Recent empirical investigations have introduced various variables affecting the environmental preservation such as FDI, globalization, institutional quality, innovation, population, and urbanization, tourism, and industrial structure [12–15] while productive capacities is little focused in the earlier literature. Economists and multilateral organizations such as UN and WTO have emphasized the importance of enhancing the productive capacity of developing economies to strengthen their financial markets and set them on the path to sustainable development. The UNCTAD has introduced a novel index of productive capacities to monitor the performance of a county and assesses strategies for improvement. UNCTAD identified 8 dimensions through which a country can enhance its productive capacity, each with its corresponding measures [7, 15–17]. Each parameter constituting the productive capacities exhibits a connection with environment. "ICT" not only influences economic growth and productivity but it also has the potential to influence the environment positively by optimizing resource utilization in various sectors, such as transport and logistics and energy, resulting in reduced energy consumption levels and associated carbon emission [17–19]. "Structural change" influences environment in a significant way. Shifting from agricultural sector to energy intensive industrial sector can heighten a country’s energy demands, potentially deteriorating environmental quality. Conversely, further progress in high technology production structure may result in reduced energy consumption, mitigating the environmental impact [20]. "Natural capital" constitutes a pivotal element in sustainable development and productivity growth [21]. Consequently, the quality of natural capital has potential to influence environment. "Human capital" exerts a profound influence on productivity of a country, and its impact extends directly and indirectly to economic growth of a country. In the early stages, an increase in human capital may lead to elevated use of nonrenewable resource and pollute the environment [22]. However, upon surpassing a certain threshold, further development of human capital fosters environmental awareness and encourages the adoption of environment friendly technologies [23] which leads to reduced carbon emission and more efficient utilization of resources [24]. "Energy" is intensely used for production purpose in economically weak countries. Limited access to energy constrains the export capacity, competitiveness, and production capabilities of a country [16, 25, 26]. Therefore, energy performance stands as a pivotal element in fostering inclusive and sustainable economic growth [27]. Enhanced energy efficiency leads to reduced energy consumption and decreased environmental deterioration [28]. Transportation generate carbon emission, contributing to approximately 18% of global carbon emissions in 2022 [29]. Due to its reliance on fossil fuel, the transport sector possesses the potential to significantly exacerbate environmental pollution [30]. "The private sector" plays a substantial role in shaping the productive capacity of a country, with certain authors asserting that the private sector utilizes resources more efficiently compared to the public sector [14, 25, 31]. Nevertheless, this perspective is contested by other authors who emphasize environmental concerns, as the private sector grapples with aligning the interests of its private stakeholders with the preservation of public environmental quality [32, 33]. "Institutions" encompass a set of formal and informal regulations. Poor institutional quality hampers the development of least developed economies by limiting the productive capacity and obstructs realization of their economic potential [34, 35]. Conversely, robust institutional quality can enhance efficiency and the enforceability of environmental regulations, thus reducing carbon emissions [36].

RETRACTED

The Belt and Road Initiative (BRI) is primarily aimed at achieving economic integration of China with the Asia Pacific, Europe, and the surrounding regions [37]. The BRI encompasses a vast network, spanning 65 nations and representing 64% of the global population, 39% of the world’s land area, 35% of international trade, and 30% of the global GDP [38, 39]. Fig 2 shows the Chinese investment in the BRI with respect to its region.

**Fig 2:** Chinese BRI investment 2020 by region. Source: Green BRI center, (https://greenfdc.org/china-belt-and-road-initiative-bri-investment-report-2020/).

Since the launch of the BRI in 2013, Chinese Outward Foreign Direct Investment has surged by 30% across BRI region. Many countries hosting BRI projects are developing economies actively seeking FDI to enhance employment, productivity, infrastructure, and overall development [40]. Decision-makers in these developing nations prioritize FDI as a means of harnessing technology spillovers [41]. Additionally, in line with the Kyoto Protocol, FDI is regarded as a critical source of capital inflow that aids the economic growth of developing nations while narrowing the gap in technical capabilities compared to more developed countries [26]. The Pollution-Haven Hypothesis (PHH) marked a turning point in the establishment of stringent environmental protection regulations in trade agreements and FDI. Consequently, multinational corporations, in pursuit of trade liberalization and economic development, began relocating the production of environmentally detrimental goods from developed countries to emerging and underdeveloped economies [23, 42–44]. This often entailed the transfer of outdated and polluting technologies. A body of research, exemplified by studies conducted by Kahouli and Omri [45] and Grossman and Krueger [46], delved into the factors underpinning trade liberalization and FDI and their implications on environment through capital and technology transfers from developed to developing economies, consistent with the Pollution Haven Hypothesis [47]. Conversely, this economic integration facilitated opportunities to receive capital and new technology from more developed nations. These technologies were deployed to enhance and replace outdated, environmentally harmful technologies. The result was a reduction in carbon emissions, contributing to both economic growth and a shift in the perception of the environment’s significance in economic development. This perspective aligns with the "pollution halo" hypothesis [48].

While carbon emissions have received extensive attention in the literature, there remains a scarcity of estimates regarding the impact of productive capacities, energy poverty, institutional quality, and urbanization on carbon emissions, particularly within Belt and Road Initiative countries. To address this knowledge gap, a panel data set encompassing 52 BRI countries covering time span from 2001–2022 was employed to empirically assess the influence of productive capacities, urbanization, energy poverty, and institutional quality on carbon emissions. Various econometric techniques, including OLS, FE, differencing GMM, system GMM, and CS-ARDL were used to analyze the dynamic connections between these variables and carbon emissions. These techniques are particularly effective in handling endogeneity issues, thus producing consistent and efficient parameter estimates. Consequently, this research provides precise and well-founded policy recommendations for mitigating carbon emissions in BRI countries.

RETRACTED

Studying the impact of productive capacities, energy poverty, FDI, urbanization and economic growth on carbon emissions in the BRI countries is of great significance for several reasons. Firstly, BRI countries collectively account for a significant portion of global carbon emissions. These countries are often characterized by rapid increasing productive capacities, urbanization, FDI and economic growth, which can lead to increased CO2 emissions [7]. Studying the impact of these factors can help identify strategies to mitigate CO2 emission. Secondly, understanding the impact of these factors on carbon emissions allows policymakers to maintain a balance between environmental sustainability and development. It’s essential to ensure that economic growth is decoupled from rising emissions. Moreover, it helps in designing effective policies and regulations that encourage cleaner production processes, the adoption of renewable energy source, and environmentally responsible financial practices. Thirdly, BRI is a massive infrastructure development project spanning multiple countries [25]. By studying the impact on carbon emissions, it is possible to promote sustainable infrastructure practices, emphasizing energy efficiency and low-carbon technologies. Moreover, this study also explores the pollution halo impact in context of BRI countries so stakeholders will be able to realize the importance of FDI for environmental preservation. Lastly, many BRI countries have made commitments to reduce carbon emissions as part of international climate agreements. Research on productive capacities, renewable energy, and FDI can help these countries meet their climate targets while balancing economic development.

RETRACTED

## 2. Theoretical foundations

This study has objective to determine the impact of productive capacities, energy poverty, urbanization, institutional quality and FDI in BRI countries. The productive capacities is a novel dimension which is hardly explored in earlier literature. The relation between carbon emissions and the productive capacities can be understood through economic and environmental theories. The productive capacities index “typically measures a country’s ability to produce goods and services efficiently” [7]. The Solow Growth Model and other growth theories provide a theoretical foundation for understanding the relationship. According to these theories, growth is driven by labor, capital, and technology [19]. An increase in productive capacities, driven by technological progress, can lead to economic growth. As economies grow, they consume more energy and resources, leading to higher carbon emissions [4, 32]. The Kuznets Curve theory also suggests that as countries develop, their income level and environmental quality exhibit an inverted U-shaped relationship [5, 49]. Initially, pollution and carbon emissions tend to increase, but beyond a certain income threshold, they start to decrease [2]. This theory implies that when a country’s productive capacities index is low, it may be at a stage where economic activities are less efficient and more carbon-intensive [50]. As the productive capacities rise, economies may shift toward more sustainable production process, potentially reducing CO2 emissions [32]. Decoupling economic growth and emissions theory is of view that economies can decouple economic growth from carbon emissions through technological advancements and policy measures. As productive capacities increase, economies transit to more energy efficient and environment friendly production method [44].

FDI brings advanced technologies and management practices to host countries [22]. If these technologies are cleaner and more energy-efficient, they can contribute to a reduction in CO2 emissions [25]. Technology transfer and technological upgrading associated with FDI can lead to the adoption of more sustainable and environmentally friendly production processes [12]. FDI encourages a shift towards cleaner and less carbon-intensive industries. As BRI countries attract investments, there may be opportunities to develop and prioritize industries that are more sustainable and have lower carbon footprints, contributing to a reduction in overall CO2 emissions [31]. Multinational corporations from countries with stringent environmental standards invest to comply with global sustainability requirements [5]. These companies may bring cleaner technologies and practices, helping to mitigate CO2 emissions in the host countries [4]. Moreover, FDI leads to improvements in energy efficiency within industries. Investments in energy-efficient technologies and processes may result in lower energy consumption and, consequently, reduced CO2 emissions per unit of output [37]. In addition, FDI can stimulate innovation and research and development activities in BRI countries. This can lead to the development and adoption of new technologies that are environmentally friendly, contributing to a decrease in CO2 emissions [43]. FDI often involves infrastructure development. If this development includes investments in sustainable and green infrastructure, it can contribute to reducing CO2 emissions associated with transportation and urbanization [36].

RETRACTED

The theoretical foundation for using renewable energy to reduce carbon emissions lies in its potential to replace fossil fuel in various sectors, like electricity generation, heat production, and transportation [51]. By substituting fossil fuels with renewable energy, it is possible to reduce CO2 emissions [23, 31]. Renewable energy is derived from organic materials and it can be harnessed in various forms, such as biofuels and biogas [32]. Renewable energy has the potential to decrease CO2 emission by displacing fossil fuels. However, the actual impact on emissions depends on factors such as sustainable management, technology efficiency, and regional considerations, making it important to carefully assess and manage the carbon footprint associated with biomass energy production and utilization [7].

The level of environmental pollution is significantly influenced by economic or income growth, as highlighted in studies [19, 23, 46]. These studies argue that the disparities in variables impacting environmental pollution are closely linked to development level. To gain a better understanding of this relationship, researchers have conducted Environmental Kuznets curve (EKC) hypothesis tests. It posits that economic activities contribute to short-term environmental pollution (supporting the "pollution heaven" hypothesis) while concurrently leading to reduced environmental pollution in the long term (supporting the "pollution halo" concept). In simpler terms, environmental pollution increases with rising income per capita up to a certain point, beyond which an inverse relationship emerges between income and declining environmental [32, 49–51].

A substantial body of research has presented compelling evidence supporting the assertion that urbanization significantly impacts carbon emissions [9, 12, 27, 52, 53]. Activities such as vehicular transportation, indoor climate regulation, and electricity consumption contribute to increased carbon emissions. Notably, urbanization drives alteration in land use pattern, encompassing deforestation, and reduction of green spaces, exacerbating carbon emission into the atmosphere [54]. To mitigate the impact of urbanization on carbon emission, the promotion of sustainable urban development practices emerges as a promising strategy. This approach encompasses the implementation of various measures, including the enhancement of public transportation, the advocacy for the adoption of renewable energy sources, and the creation of green spaces and urban agriculture. These initiatives are proposed to effectively address environmental concerns by reducing waste and pollution while safeguarding finite natural resources [28, 55]. Energy poverty carries significant repercussions for environmental health, intertwining with factors such as biodiversity loss, deforestation, climate change, and restricted access to clean environment [56, 57]. Tackling energy poverty is paramount not only to increase the quality of life for those deprived of modern energy services but also to protect the natural environment and foster sustainable development [58].

RETRACTED

## 3. Literature review

Within the existing literature, the studies investigated the environmental consequences of various factors such as economic complexity, GDP, transportation, urbanization, export diversification, FDI, renewable energy, population growth, productive capacities, industrialization, and human capital. Table 1 offers a summary of key studies in the literature of environmental economics. None of these studies have undertaken a comprehensive examination of productive capacities for environmental preservation.

**Table 1:** Related literature.

Study	Sample	Time Period	Main Variable	Indicator of Environment	Methodology	Findings
Caglar & Mert [1]	Top 5 emitting countries	1965–2020	Carbon hysteresis hypothesis	CO2 emission	Unit Root tests	Validity of hypothesis
Caglar et al. [2]	BRICS	1990–2018	Competitive Industrial Performance	Load Capacity factor	CUP-FM CUP-BC	Positive relationship
Caglar [3]	UK	1974–2020	Nuclear energy	CO2 emission	NARDL	Negative relationship
Caglar et al. [4]	EU	1995–2018	Renewable energy	Load Capacity factor	CUP-FM CUP-BC	Positive relationship
Caglar & Yavuz [5]	EU	1995–2018	Environmental protection expenditures	Load Capacity factor	CS-ARDL	Positive relationship
Caglar & Askin [6]	Top 10 CIP Economies	1990–2018	Competitive Industrial performance	CO2 emission, Load Capacity factor	Panel Techniques	Negative relationship
Madni [7]	42 BRI countries	2000–2018	Productive capacities	Ecological Footprint	CC-EMG	Negative relationship
Ahmed et al. [31]	G7 Countries	1985 to 2017	Economic Complexity	Ecological Footprint	CUP-FM	Negative relationship
Hassan et al. [19]	BRICS	1989–2016	Energy Poverty	CO2	CC-EMG	Positive relationship
Adebayo et al. [32]	Turkey	1965 to 2019	Structural Changes	CO2	NARDL	Negative relationship
Anwar et al. [51]	BRI Countries	1986 to 2017	Industrialization	CO2	ARDL	Negative relationship
Can & Gozgor [52]	France	1964–2014	Economic Complexity	CO2 Emissions	DOLS	Negative relationship
Neagu & Teodoru [53]	European Union	1995–2016	Economic Complexity	GHG emission	FMOLS	Positive relationship
He et al. [54]	Top 10 Energy transition countries	1990 to 2018	Economic Complexity	CO2	CS-ARDL	Negative relationship
Zhang & Liu [28]	China	2000–2010	ICT	CO2	AMG	Positive relationship
Sun et al. [55]	N-11	1990–2018	Institutional quality	Ecological Footprint	CS-ARDL	Negative relationship
Wu & Madni [56]	33 BRI Countries	1986–2018	Institutional quality	CO2	Threshold Regression	Negative relationship
Zhao & Madni [57]	122 Countries	1996–2020	Institutional Reforms	CO2	DID	Negative relationship
Christoforidis & Katrakilids [58]	OECD countries	1984 to 2016	Institutions	Ecological Footprint	DOLS-MG	Negative relationship
Sahoo & Sethi [59]	36 Developing Countries	1990 to 2016	Natural Resources	Ecological Footprint	AMG	Negative relationship
Haseeb et al. [60]	BRICS	1994 to 2014	ICT	CO2	DSUR	Negative relationship
Godil et al. [61]	USA	2000–2019	Transportation	CO2	QARDL	Negative relationship
Saboori et al. [62]	OECD Countries	1960 to 2008	Transportation	CO2	FMOLS	Positive relationship
Peng et al. [63]	BRICS	1992 to 2018	Economic Complexity	CO2	CUP-FM	Negative relationship
Martins et al. [64]	7 complex economies	1993 to 2018	Economic Complexity	CO2	CS-ARDL	Positive relationship
Khan & Hou [65]	38 Countries	1995–2018	Energy Consumption	Ecological Footprint	FMOLS	Positive relationship
Sharif et al. [66]	74 Countries	1990 to 2015	Renewable energy consumption	CO2	FMOLS	Negative relationship

RETRACTED

## 4. Methodology

In the present study, the following regression is formulated.


$${\text{CRE}}_{\text{it}}=\alpha_{0}+\alpha_{1}{\text{PRC}}_{\text{it}}+\alpha_{2}{\text{EGP}}_{\text{it}}+\alpha_{3}{\text{URB}}_{\text{it}}+\alpha_{4}{\text{IQL}}_{\text{it}}+\alpha_{\text{n}}{\text{Z}}_{\text{it}}+\epsilon_{\text{it}}$$

The above model explores the connection between carbon emissions and various independent variables. The model includes productive capacities (PRC), energy poverty (EGP), urbanization (URB), institutional quality (IQL), and Z is set of control variables. The theoretical relationship of these variables have been explained in the earlier section 2. The description of variables and sources of data are shown in the following Table 2.

**Table 2:** Description of variables and sources.

Variable	Description	Source
Carbon Emissions	CO2 emissions metric tons per capita	WDI
Productive Capacities	Productive Capacities Index	UNCTAD
Energy Poverty	Proportion of individuals have not access to energy infrastructure	WDI
Urbanization	Urbanization (% of total population)	WDI
Institutional Quality	Governance Variable	WGI
Foreign Direct Investment	FDI as percentage of GDP	WDI
Renewable Energy	Percentage of renewable energy out of total energy	WDI
Economic Growth	GDP per capita	WDI

This study commenced by conducting panel unit root tests to assess the data’s stationarity. After these initial tests, the formal analysis was carried out using OLS, FE, DGMM, SGMM, CS-ARDL. Ordinary Least Squares (OLS) is widely used because it has closed-form solutions for estimating the parameters, making it computationally efficient [21]. OLS is a method used in regression analysis to estimate the parameters of a linear regression model. It is a way that minimizes the sum of the squared differences between the observed values of the dependent variable and the values predicted by the model [35]. To estimate the parameters, specify a linear relationship between the dependent and independent variables. Then minimize the sum of the squared differences between the observed values of the dependent variable and the values predicted by the model. This is done by adjusting the model parameters until the sum of squared residuals is minimized [46]. Once the model parameters are determined, they provide the estimated values for the slope and intercept of the regression line.

The fixed effects (FE) technique is used to control for unobserved, time-invariant factors that may be influencing the dependent variable. Fixed effects models are particularly useful when there are concerns about unobserved heterogeneity among the subjects in a panel dataset, and where observations are made on the same individuals, entities, or groups over multiple time periods [50]. The goal of fixed effects is to account for individual-specific characteristics that do not change over time but may still affect the dependent variable. In a regression model with fixed effects, the individual-specific effects are included as fixed parameters [37]. Least squares or maximum likelihood, are used to estimate the coefficients and the fixed effects. The fixed effects capture the individual-specific characteristics that do not vary over time. By including fixed effects in the model, influence of time-invariant factors is controlled and focus on estimating the effects of the time-varying explanatory variables.

The Generalized Method of Moments (GMM) is a broader and more general statistical framework compared to OLS. GMM is widely used for estimating parameters in econometric models and addressing issues such as endogeneity and instrument variable problems [7]. GMM estimates parameters by choosing them to satisfy a set of moment conditions [57]. These moment conditions are functions of the data and parameters, and the estimation process involves choosing parameters that make these conditions as close to zero as possible. It provides estimates that are asymptotically efficient and can be more efficient than OLS, especially in the presence of heteroscedasticity and endogeneity [46].

RETRACTED

System GMM is an extension of the GMM that addresses some of the limitations of the standard GMM, particularly when dealing with dynamic panel data models, where both lagged values of the dependent variable and predetermined variables are included as explanatory variables [52]. These models are characterized by the presence of unobserved individual effects and endogeneity. It is widely employed in econometric studies to handle endogeneity, heteroscedasticity, and unobserved individual effects [59]. Endogeneity is a common issue due to the correlation between the lagged dependent variable and the error term so it addresses by using lagged levels of the endogenous variable as instruments. It typically involves a two-step estimation procedure. In the first step, the system is differenced to eliminate individual effects, and a first-differenced GMM estimator is applied. In the second step, the first-differenced equation is used to instrument the levels equation. System GMM uses a set of instruments to construct moment conditions [62]. These instruments are typically lagged levels and first-differences of the regressors and lagged levels of the dependent variable [38]. The choice of instruments is crucial for the efficiency and consistency of the estimates. Moreover, system GMM accounts for potential autocorrelation in the differenced equation by introducing additional moment conditions based on the residuals from the differenced equation.

Regressing a Cross-Sectional Autoregressive Distributed Lag (CS-ARDL) model involves estimating the parameters that characterize the relationships between variables for each cross-sectional unit in a panel data setting [6]. The CS-ARDL model is an extension of the ARDL model to panel data. Estimation methods for panel data, such as the Fixed Effects (FE) or Random Effects (RE) methods are applied [29]. The estimation process involves obtaining estimates for the coefficients in the model. Apply panel cointegration tests to determine if there is a long-term relationship among the variables for each cross-sectional unit [53].

RETRACTED

Initially, static models such as OLS and FE were employed to address heterogeneity, enabling comparisons with prior research and serving as benchmarks against the dynamic model results. The introduction of the GMM model aimed to tackle endogeneity concerns related to the study’s variables [61]. The model’s specified instruments include the lag values of level difference equations, encompassing the horizontal equation and the first difference mean of the study variables. The over-identifying restriction tests have been replaced by the Sargan test, which confirms the alignment of the study model’s expectations. The inclusion of the first lag of carbon emissions as an independent variable helps to assess the influence of the prior year’s carbon emissions on present carbon emissions.

## 5. Results and discussion

Before commencing the formal analysis, we applied second generation unit root tests to assess stationarity. As recommended by [62], the study utilized the CADF and CIPS tests and the results for all countries and variables in the sample are presented in Table 3.

**Table 3:** Panel unit root test.

Variable	CIPS		CADF	
	Level	Difference	Level	Difference
CRE	-2.035	-3.62***	-1.29	-3.96***
PRC	-3.62	-4.51***	-2.54	-4.88***
EGP	-2.32	-3.67***	-1.95	-3.96***
URB	-2.06	-3.64***	-2.38	-3.83***
IQL	-1.35	-2.13***	-1.56	-2.63***
FDI	-3.64***	-4.58***	-2.96***	-4.72***
RNY	-1.37	-2.13***	-1.26***	-2.24***
ECG	-2.38	-3.69***	-2.15***	-3.76***

Note:

*** show significance at 1%.

The above results indicated that all the variables under examination exhibited stationarity at the level or first differences. The variables in the study were all subjected to testing at first-difference level, yielding significant results. Consistent with the outcomes of the second-generation tests, the variables in question demonstrated stationarity at either the levels or first-order differences. Following the determination of unit root status, the study assessed cross-sectional dependence. The results of the tests for cross-sectional dependence, conducted on a panel encompassing 52 BRI economies, are presented in Table 4.

**Table 4:** Cross sectional dependence.

Test	Values
Friedman’s Test	141.43***
Pesaran’s Test	35.26***
Frees’ Test	12.36

Note:

*** show significance at 1%.

These tests are conducted to determine whether there is any correlation or dependence among individual observations across the units. There are three common tests to determine the cross sectional dependence. Westerlund test is conducted to find the long run relation and results indicate the presence of long run co-integrating relationship among variables as shown in the following Table 5.

RETRACTED

**Table 5:** Panel co-integration test.

Westerlund Test	Statistics
Variance Ratio	1.88***
Pedroni Test for Co-integration	
Modified Philips-Perron t	11.77
Philips-Perron t	-6.82
Augmented Dicky-Fuller t	-7.86

Note:

*** shows significance at 1% level.

Once cross-sectional dependence is established, the estimated results obtained through various methods, including OLS, FE, DGMM, SGMM, Cross sectional augmented autoregressive distributed lag (CS-ARDL) are presented in Table 6.

**Table 6:** Estimated results.

Variables	OLS	FE	DGMM	SGMM	CS-ARDL	
					Long Run Estimates	Short Run Estimates
CRE (-1)			0.13***	0.25***		-0.31***
PRC	-0.28***	-0.19***	-0.31***	-0.29***	-0.28**	-3.62
EGP	0.13***	0.14**	0.16***	0.18***	0.13***	0.11**
URB	0.16***	0.20**	0.29***	0.09***	0.13***	0.05**
IQL	-0.08***	-0.10***	-0.12***	-0.16***	-0.16**	0.07***
FDI	-0.03**	-0.06**	-0.07***	-0.06***	-0.08**	-0.04**
RNY	-0.18***	-0.17***	-0.21***	-0.29***	-0.22**	-0.11**
ECG	-0.02	0.27***	0.06**	0.05***	0.15***	0.06**
Constant	-2.05**	1.38		-0.08	-3.62	-2.38
R2	0.52	0.55			0.58	0.66
AR 1			0.03***	-1.98***		
AR 2			-0.22***	-0.58***		
Sargan Test			11.82	14.26		

Note:

*** and ** show significance at 1% and 5% respectively.

The results indicate that productive capacities have a negative impact, suggesting that they lead to a reduction in carbon emissions. This highlights the importance of considering the productive capacities of the sample countries as a means to enhance environmental quality. Furthermore, the findings depict that all models consistently yield positive and significant impact of EGP and URB on carbon emissions. This is attributed to the fact that EGP promotes traditional energy usage, while urbanization tends to increase carbon dioxide concentration in the sample, thereby diminishing environmental quality. The ECG has substantial but negative impact on carbon emissions, indicating that it results in higher carbon dioxide emissions. Empirical analysis also reveals that RNY, IQL, and FDI play significant roles in reducing environmental pollution. Additionally, AR(1) coefficient is significant, with a p-value less than 0.01, while the AR(2) coefficient is not significant, suggesting the absence of substantial second order error autocorrelation. This result further supports the suitability and effectiveness of the DGMM and SGMM approach used in this study. The Sargan test assesses the validity of the over-identification restrictions in GMM estimation.

## 6. Discussion

The findings of this study highlight that productive capacities play a significant role in decreasing carbon emissions. Here are several ways in which productive capacities can be leveraged to reduce carbon emissions. Firstly, investment in and deploy cleaner and more energy efficient technologies in production processes reduces carbon emissions. This can include upgrading equipment, implementing energy efficient practices, and using renewable energy sources. Secondly, improving energy efficiency throughout the production process reduces the dependency on traditional energy usages. This involves reducing energy waste and optimizing the use of resources to minimize carbon emissions associated with energy consumption [19]. Thirdly, transition to renewable energy sources to power production facilities to reduce carbon emissions. This reduces reliance on fossil fuels and lowers carbon emissions associated with electricity and heat generation [41]. In summary, productive capacities can significantly decrease carbon emissions through a combination of technological advancements, efficiency improvements, and sustainable practices [47]. Businesses and industries that actively work to reduce their carbon footprint not only contribute to global efforts to combat climate change but also often find cost-saving opportunities and enhance their reputation as environmentally responsible entities [59]. The findings of this study are consistent with findings of earlier studies [8, 16, 19, 41, 47].

RETRACTED

Urbanization refers to a socioeconomic phenomenon involving the movement of people from rural areas to urban centers [35]. Over the recent years, this trend has been particularly prominent in developing countries, including those situated along the BRI route. However, rapid urbanization is often associated with negative environmental impacts, notably an increase in carbon emissions [21, 36, 52]. The relation between urbanization and carbon emissions is complex and depends on various factors, including urban planning, infrastructure, and lifestyle choices. Urban areas often have higher energy demands due to the concentration of people, businesses, and industries. Increased energy consumption, especially if sourced from fossil fuels, can lead to higher carbon emissions [36]. However, the energy efficiency of buildings and transportation systems can influence the overall emissions from urban areas [25]. Secondly, urbanization can lead to greater transportation emissions, primarily if it results in increased reliance on personal vehicles [13]. Longer commutes, traffic congestion, and inadequate public transportation infrastructure can contribute to higher carbon emissions [31]. Thirdly, urban areas generate large quantities of waste and pollution. Effective waste management and pollution control measures can mitigate the environmental impact [22]. Recycling and waste-to-energy technologies can help reduce emissions from waste. Lastly, the lifestyle choices of urban residents can affect emissions. People living in cities may have smaller living spaces and be more likely to use public transportation, but they might also engage in more consumerism and higher-density living [49]. Education and awareness campaigns can encourage sustainable consumer choices. The findings of the current study are in line with earlier studies [21, 23, 25, 36, 56].

RETRACTED

Institutional quality, which refers to the effectiveness and strength of a country’s institutions, play a crucial role in reducing carbon emissions. Strong and well-functioning institutions create an environment that fosters sustainable development and enforces regulations aimed at mitigating climate change [59]. High-quality institutions establish and enforce environmental regulations and standards. These regulations can set emission limits, promote the use of clean technologies, and require businesses to adopt practices that reduce carbon emissions [49, 67]. Secondly, strong institutions ensure that environmental regulations are effectively enforced. This discourages non-compliance and penalizes those who exceed emission limits, encouraging firms to reduce their carbon emissions [39, 68]. Institutions can offer incentives, subsidies, and support for the development and adoption of clean energy technologies, such as renewable energy sources (solar, wind, hydro, etc.) and energy-efficient solutions [44]. These policies can reduce reliance on fossil fuel and lower carbon emissions. High-quality institutions promote public participation and the activities of civil society organizations that advocate for sustainable and low-carbon policies [25]. Public pressure and advocacy can influence government decisions and corporate behavior regarding emissions reduction. These findings are in line with findings of the earlier literature [23, 25, 39, 52, 57].

Moreover, energy poverty carries adverse environmental consequences as it often leads households to rely on traditional energy sources, which are widely recognized as unsustainable [23, 69]. These traditional energy sources release substantial amounts of carbon emissions, contributing to climatic changes. In the specific context of the Belt and Road Initiative region, energy poverty exacerbates carbon emissions due to developmental constraints. The poverty experienced in these countries is compounded by lack of access to modern energy services, which hinders their ability to transition to cleaner and more sustainable energy. The findings presented here align with the conclusions of earlier studies [25, 31, 57, 61].

RETRACTED

The discussion surrounding the potential mitigating effects of RNY on carbon emissions suggests that nations have the capacity to reduce their carbon emissions by increasing their reliance on renewable energy sources [59]. These renewable energy sources possess the advantage of generating energy without emitting greenhouse gases. In addition, observed negative impact of foreign direct investment on carbon emissions in Belt and Road Initiative countries imply a pollution halo effect. FDI potentially lead to decreased carbon emissions by adopting environmentally friendly technologies and practices. Other factors may contribute to the mentioned adverse consequences, suggesting that the relationship between FDI and carbon emissions is more intricate than a straightforward linear association [52, 58].

## 7. Conclusions

The BRI represents one of the transformative economic development projects in the contemporary world. As BRI countries continue to experience rapid industrialization and growth, it becomes increasingly important to analyze the impact of productive capacities, FDI, renewable energy, energy poverty, urbanization, and economic growth on Carbon emissions. This research provides valuable insights into the link between carbon emissions and factors such as productive capacities, urbanization, institutional quality, and energy poverty in BRI countries. Through the analysis of panel data of 52 BRI countries from 2001–2022, this study employed various models, including OLS, FE, DGMM, SGMM, and CS-ARDL to determine the impact of these diverse factors on carbon emissions. Our analysis has explored several key findings, each of which carries significant implications for sustainable development, environmental conservation, and global climate change mitigation. It is evident that the expansion of productive capacities in BRI countries has been accompanied by reduced carbon emissions. The findings on how productive capacities reduce carbon emission revolves around the notion that enhanced productive capabilities can lead to reduce carbon emissions through increased energy efficiency, technological advancements, and sustainable practices. Moreover, institutional quality, renewable energy and FDI reduce CO2 emissions proving pollution halo impact. In addition, energy poverty, urbanization, and economic growth have positive impact on CO2 emissions in the BRI region.

Based on these empirical findings, the following policy recommendations are put forth for the consideration of stakeholders and governments in BRI countries. Firstly, it is evident that enhancing a country’s productive capacity plays a significant role in reducing carbon emissions. As the PCI index comprises eight main components, improvements in each of these areas can collectively contribute to reducing carbon emissions. Thus, the study proposes the following policies: Encourage the widespread adoption of ICT to optimize management planning, supply chain logistics, and trade. Leveraging the internet’s global reach can enhance information exchange, leading to greater energy efficiency, reduced time wastage, and lower environmental pollution. Policymakers should support investments in ICT. To decarbonize the transportation sector, clean technologies should be supported through tax incentives and subsidies, making them more competitive and reducing environmental pollution. Governments can allocate budgets to bolster the transportation industry’s efforts to adopt cleaner technologies. Collaboration between the public and private sectors is essential to combat environmental pollution. Developing countries should prioritize improving institutional quality as a top national priority for reducing carbon emissions. Strict enforcement of environmental laws, restructuring of environmental protection mechanisms, and an emphasis on enhancing institutional performance are crucial.

RETRACTED

Policymakers should prioritize providing affordable and sustainable energy to public. This can be achieved by implementing solar or wind energy systems and programs to enhance energy efficiency. Encourage companies to adopt cleaner production technologies through mechanisms like tax breaks or subsidies. Policymakers should focus on balancing economic development with environmental preservation by implementing rigorous environmental regulations, advocating for circular economy principles, and incorporating eco-friendly technologies. Dedicate resources to research and development initiatives aimed at fostering innovation in sustainable practices. Although the findings of this study hold significance for policymakers, it’s crucial to recognize its constraints and identify avenues for further research. Some limitations and potential areas for future research encompass that future research can consider additional indicators of environmental instability, such as the ecological footprint, to provide a more comprehensive picture of the impact of pollution. Expanding the scope of the study to include other regions and economies beyond the 52 BRI countries could offer further insights into the relationship between various factors and environmental pollution. This would be particularly valuable with access to larger datasets. By addressing these limitations and extending the study to encompass a wider array of factors and regions, researchers can contribute to a more holistic understanding of this intricate relationship.

RETRACTED

## Abbreviations

BRI: Belt and Road Initiative
CS-ARDL: Cross sectional augmented autoregressive distributed lag
DGMM: Difference GMM
FE: Fixed Effect
GMM: Generalized Method of Moments
OLS: Ordinary Least Square
SGMM: System GMM
UN: United Nations
UNCTAD: UN Conference on Trade and Development
WTO: World Trade Organization

## References

[1] CaglarA.E.; MertM. Carbon hysteresis hypothesis as a new approach to emission behavior: A case of top five emitters. Gondwana Research. 2022, 109, 171–182.

[2] CaglarA.E.; DaştanM., MehmoodU. et al. Assessing the connection between competitive industrial performance on load capacity factor within the LCC framework: Implications for sustainable policy in BRICS economies. Environ Sci Pollut Res. 2023. doi: 10.1007/s11356-023-29178-1 37608171

[3] CaglarA.E. Can nuclear energy technology budgets pave the way for a transition toward low-carbon economy: Insights from the United Kingdom. Sustainable Development. 2022, 31(12), 1–13.

[4] CaglarA.E.; DaştanM.; BulutE.; MarangozC. Evaluating a pathway for environmental sustainability: The role of competitive industrial performance and renewable energy consumption in European countries. Sustainable Development. 2023. doi: 10.1002/sd.2755

[5] CaglarA.E.; YavuzE. The role of environmental protection expenditures and renewable energy consumption in the context of ecological challenges: Insights from the European Union with the novel panel econometric approach. Journal of Environmental Management. 2023, 331, 117317. doi: 10.1016/j.jenvman.2023.117317 36669312

[6] CaglarA.E.; AskinB.E. A path towards green revolution: How do competitive industrial performance and renewable energy consumption influence environmental quality indicators? Renewable Energy. 2023, 205, 273–280.

[7] MadniG.R. Meditation for role of productive capacities and green investment on ecological footprint in BRI countries. Environ Sci Pollut Res. 2023, 30(28):72308–72318. doi: 10.1007/s11356-023-27478-0 37170048

[8] MertM.; CaglarA.E. Testing pollution haven and pollution halo hypotheses for Turkey: A new perspective. Environmental Science and Pollution Research. 2020, 27, 32933–32943. doi: 10.1007/s11356-020-09469-7 32524397 PMC7283984

[9] BarkatK.; AlsamaraM.; MimouniK. Can remittances alleviate energy poverty in developing countries? New evidence from panel data. Energy Econ. 2023, 119:106527.

[10] ChienF.; HsuC.C.; OzturkI.; SharifA.; SadiqM. The role of renewable energy and urbanization towards greenhouse gas emission in top Asian countries: evidence from advance panel estimations. Renew Energy. 2022, 186:207–216.

[11] SalamM.; XuY. Trade openness and environment: a panel data analysis for 88 selected BRI countries. Environmental Science and Pollution Research. 2022, 29:23249–23263. doi: 10.1007/s11356-021-17037-w 34800274

RETRACTED

[12] MurshedM.; ApergisN.; AlamM.S.; KhanU.; MahmudS. The impacts of renewable energy, financial inclusivity, globalization, economic growth, and urbanization on carbon productivity: evidence from net moderation and mediation effects of energy efficiency gains. Renew Energy. 2022, 196:824–838.

[13] ZhaoJ.; JiangQ.; DongX.; DongK. Assessing energy poverty and its effect on CO2 emissions: the case of China. Energy Econ. 2021, 97:105191.

[14] WangQ.; WangL. How does trade openness impact carbon intensity? J. Cleaner Prod. 2021, 295 (1), 126370.

[15] UNCTAD. UNCTAD productive capacities index: methodological approach and results, 2021, 63. https://unctad.org/system/files/official-document/aldc2020d3_en.pdf.

[16] UNCTADSTAT. United Nations Conference on Trade and Development Data Center. 2021. https://unctadstat.unctad.org/wds/Table Viewer/tableView.aspx?ReportId=199270

[17] DoğanB.; SabooriB.; CanM. Does economic complexity matter for environmental degradation? An empirical analysis for different stages of development. Environ Sci Pollut Res. 2019, 26(31):31900–31912. doi: 10.1007/s11356-019-06333-1 31489548

[18] KurniawanR.; ManagiS. Linking wealth and productivity of natural capital for 140 countries between 1990 and 2014. Soc Indic Res. 2019, 141(1):443–462.

[19] HassanS.T.; BatoolB.; ZhuB.; KhanI. Environmental complexity of globalization, education, and income inequalities: new insights of energy poverty. J Clean Prod. 2022, 340:130735.

[20] ZhangS.; LiZ.; NingX.; LiL. Gauging the impacts of urbanization on CO2 emissions from the construction industry: evidence from China. J Environ Manag. 2021, 288:112440. doi: 10.1016/j.jenvman.2021.112440 33831637

[21] QureshiS.; NajjarL. Information and communications technology use and income growth: evidence of the multiplier effect in very small island states. Inf Technol Dev. 2017, 23(2):212–234.

[22] ChattiW. Moving towards environmental sustainability: information and communication technology (ICT), freight transport, and CO2 emissions. Heliyon. 2021, 7(10): e08190. doi: 10.1016/j.heliyon.2021.e08190 34729432 PMC8546415

[23] WangH.; WeiW. Coordinating technological progress and environmental regulation in CO2 mitigation: the optimal levels for OECD countries & emerging economies. Energy Economics. 2020, 87:104510.

[24] YuanC.; LiuS.; FangZ.; WuJ. Research on the energy-saving effect of energy policies in China: 1982–2006. Energy Policy. 2009, 37(7):2475–2480.

[25] CanB.; CanM. Examining the relationship between knowledge and well-being as values of a society. Regulating Human Rights Soc Secur Socio-Econ Struct Global Perspect. 2022, 211–226. IGI Global.

RETRACTED

[26] KhanS.; YahongW. Income inequality, ecological footprint, and carbon dioxide emissions in Asian developing economies: what effects what and how? Environ Sci Pollut Res. 2022, 29:24660–24671.10.1007/s11356-021-17582-434826073

[27] DemissewB.S.; KotoszB. Testing the environmental Kuznets curve hypothesis: an empirical study for East African countries. Int J Environ Stud. 2020, 77(4):636–654.

[28] ZhangC.; LiuC. The impact of ICT industry on CO2 emissions: a regional analysis in China. Renew Sustain Energy Rev. 2015, 44:12–19.

[29] International Energy Agency. Electricity market report–January 2022. IEA, Paris. 2022. https://www.iea.org/reports/electricitymarket-report-January-2022

[30] ZhaoJ.; ShahbazM.; DongK. How does energy poverty eradication promote green growth in China? The role of technological innovation. Technol Forecast Soc Chang. 2022,175:121384.

[31] AhmedZ.; AdebayoT.S.; UdembaE.N.; MurshedM.; KirikkaleliD. Effects of economic complexity, economic growth, and renewable energy technology budgets on ecological footprint: the role of democratic accountability. Environ Sci Pollut Res. 2022, 29(17):24925–24940. doi: 10.1007/s11356-021-17673-2 34826087

[32] AdebayoT.S.; OladipupoS.D.; RjoubH.; KirikkaleliD.; AdesholaI. Asymmetric effect of structural change and renewable energy consumption on carbon emissions: designing an SDG framework for Turkey. Environ Dev Sustain. 2022, 1–29. doi: 10.1007/s10668-021-02065-w 35002481 PMC8723907

[33] SantosG. Road transport and CO2 emissions: what are the challenges? Transp Policy. 2017, 59:71–74.

[34] HancockC.; KingoL.; RaynaudO.The private sector, international development and NCDs. Glob Health. 2011, 7(1):23.10.1186/1744-8603-7-23PMC316318321798001

[35] TalukdarD.; MeisnerC.M. Does the private sector help or hurt the environment? Evidence from carbon dioxide pollution in developing countries. World Dev. 2001, 29(5):827–840.

[36] RashedA.H.; ShahA. The role of private sector in the implementation of sustainable development goals. Environ Dev Sustain. 2021, 23(3):2931–2948.

[37] CassonM.C.; DellaG.M.; KambhampatiU.S. Formal and ınformal ınstitutions and development. World Dev. 2010, 38(2):137–141.

[38] BhattacharyaM.; AwaworyiC.S.; ParamatiS.R. The dynamic impact of renewable energy and institutions on economic output and CO 2 emissions across regions. Renewable Energy. 2017, 111:157–167.

[39] LeeH.S.; MoseykinY.N.; ChernikovS.U. Sustainable relationship between FDI, R&D, and CO2 emissions in emerging markets: an empirical analysis of BRICS countries. Russ J Econ. 2021, 7:297–312.

RETRACTED

[40] RehmanA.; MaH.; OzturkI.; UlucakR. Sustainable development and pollution: the effects of CO2 emission on population growth, food production, economic development, and energy consumption in Pakistan. Environ Sci Pollut Res. 2021, 1–12. doi: 10.1007/s11356-021-16998-2 34661835

[41] HussainM.N.; LiZ.; SattarA.; IlyasM. Evaluating the impact of energy and environment on economic growth in BRI countries. Energy Environment. 2022. 0958305X211073805.

[42] HailuZ.A. Impact of foreign direct investment on trade of African countries. International Journal of Economics and Finance. 2010, 2(3), 122–133.

[43] GillF.L.; ViswanathanK.K.; KarimM.Z.A. The critical review of the pollution haven hypothesis. International Journal of Energy Economics and Policy. 2018, 8(1), 167–174.

[44] CopelandB.; TaylorM.S. North-South trade and the environment. The Quarterly Journal of Economics. 1994, 109(3), 755–787.

[45] KahouliB.; OmriA. Foreign direct investment, foreign trade and environment: New evidence from simultaneous-equation system of gravity models. Research in International Business and Finance. 2017, 42, 353–364.

[46] Grossman, G.M.; Krueger, A.B. Environmental Impacts of a North American Free Trade Agreement. United States: NBER Working Paper. 1991, 3914.

[47] ZakaryaG.Y.; MostefaB.; AbbesS.M.; SeghirG.M. Factors affecting CO2 emissions in the BRICS countries: A panel data analysis. Procedia economics and finance. International Journal of Energy Economics and Policy. 2015, 8(5), 114–125.

[48] FrankelJ.; RoseA. An estimate of the effect of common currencies on trade and income. The Quarterly Journal of Economics. 2002, 117(2), 437–466.

[49] GrossmanG.; KruegerA. Environmental ımpacts of a North American Free Trade Agreement. National Bureau of economic research, Cambridge, MA. 1991. doi: 10.3386/w3914

[50] AminM.; ZhouS.; SafiA. The nexus between consumption based carbon emissions, trade, eco-innovation, and energy productivity: empirical evidence from N-11 economies. Environ Sci Pollut Res. 2022, 29(26):39239–39248. doi: 10.1007/s11356-021-18327-z 35098468

[51] AnwarA.; AhmadN.; MadniG.R. Industrialization, freight transport and environmental quality: evidence from belt and road initiative economies. Environmental Sci Pollu Res. 2020, 27:7053–70. doi: 10.1007/s11356-019-07255-8 31879891

[52] CanM.; GozgorG. The impact of economic complexity on carbon emissions: evidence from France. Environ Sci Pollut Res. 2017, 24(19):16364–16370.10.1007/s11356-017-9219-728547378

[53] NeaguO.; TeodoruM.C. The relationship between economic complexity, energy consumption structure and greenhouse gas emission: heterogeneous panel evidence from the EU countries. Sustainability. 2019. doi: 10.3390/su11020497

RETRACTED

[54] HeK.; RamzanM.; AwosusiA.A.; AhmedZ.; AhmadM.; AltuntaşM. Does globalization moderate the effect of economic complexity on CO2 emissions? evidence from the top 10 energy transition economies. Front Environ Sci. 2021, 9:778088.

[55] SunY.; TianW.; MehmoodU.; ZhangX.; TariqS. How do natural resources, urbanization, and institutional quality meet with ecological footprints in the presence of income inequality and human capital in the next eleven countries? Resources Policy. 2023, 1; 85:104007.

[56] WuQ.; MadniG.R. Environmental protection in selected one belt one road economies through institutional quality: Prospering transportation and industrialization. PloS ONE. 2021, 14; 16(1): e0240851. doi: 10.1371/journal.pone.0240851 33444315 PMC7808598

[57] ZhaoJ.; MadniG.R. The impact of economic and political reforms on environmental performance in developing countries. PLoS ONE. 2021, 16(10): e0257631. doi: 10.1371/journal.pone.0257631 34610016 PMC8491874

[58] ChristoforidisT.; KatrakilidisC. The dynamic role of institutional quality, renewable and non-renewable energy on the ecological footprint of OECD countries: do institutions and renewables function as leverage points for environmental sustainability? Environ Sci Pollut Res. 2021, 28(38): 53888–53907. doi: 10.1007/s11356-021-13877-8 34037934

[59] SahooM.; SethiN. The intermittent effects of renewable energy on ecological footprint: evidence from developing countries. Environmental Science and Pollution Research. 2021, 28(40):56401–17. doi: 10.1007/s11356-021-14600-3 34053045

[60] HaseebA.; XiaE.; SaudS.; AhmadA.; KhurshidH. Does information and communication technologies improve environmental quality in the era of globalization? An empirical analysis. Environ Sci Pollut Res. 2019, 26(9):8594–8608. doi: 10.1007/s11356-019-04296-x 30710332

[61] GodilD.I.; YuZ.; SharifA.; UsmanR.; KhanS.A.R. Investigate the role of technology innovation and renewable energy in reducing transport sector CO2 emission in China: a path toward sustainable development. Sustain Dev. 2021, 29(4):694–707.

[62] SabooriB.; SapriM.; BabaM. Economic growth, energy consumption and CO2 emissions in OECD (Organization for Economic Co-operation and Development)’s transport sector: a fully modified bi-directional relationship approach. Energy. 2014, 66:150–161.

[63] PengG.; MengF.; AhmedZ.; AhmadM.; KurbonovK. Economic growth, technology, and CO2 emissions in BRICS: investigating the non-linear impacts of economic complexity. Environ Sci Pollut Res. 2022, 1–12. doi: 10.1007/s11356-022-20647-7 35526204

[64] MartinsJ.M.; AdebayoT.S.; MataM.N.; OladipupoS.D.; AdesholaI.; AhmedZ.; et al. Modeling the relationship between economic complexity and environmental degradation: evidence from top seven economic complexity countries. Front Environ Sci. 2021, 9:1–12.

RETRACTED

[65] KhanI.; HouF. The dynamic links among energy consumption, tourism growth, and the ecological footprint: the role of environmental quality in 38 IEA countries. Environ Sci Pollut Res. 2021, 28(5): 5049–5062. doi: 10.1007/s11356-020-10861-6 32951171 PMC7502029

[66] SharifA.; RazaS.A.; OzturkI.; AfshanS. The dynamic relationship of renewable and nonrenewable energy consumption with carbon emission: a global study with the application of heterogeneous panel estimations. Renew Energy. 2019, 133:685–691.

[67] QianC.; MadniG.R. Encirclement of Natural Resources, Green Investment, and Economic Complexity for Mitigation of Ecological Footprints in BRI Countries. Sustainability. 2022, 14, 15269.

[68] MadniG. R.; AnwarM. A.; AhmadN. Socio-economic Determinants of Environmental Performance in Developing Countries. Journal of Knowledge Economy. 2021, 13, 1157–1168.

[69] WangC.; CardanP. W.; LiuG.; MadniG.R. Social and economic factors responsible for environmental performance: A global analysis. PLOS ONE. 2020, 15(8): e0237597. doi: 10.1371/journal.pone.0237597 32853232 PMC7451562

